The article "First Branchial Cleft Anomalies: Awareness Is Key" was published in 2021. Journal: Cureus.

# First Branchial Cleft Anomalies: Awareness Is Key

**DOI:** 10.7759/cureus.20655

**Published:** 2021-12-24

**Authors:** Javier Ash, Oliver H Sanders, Tarik Abed, Jonathan Philpott

**Affiliations:** 1 Otolaryngology, Southend University Hospital, Southend-on-Sea, GBR

**Keywords:** poncet's triangle, peri-auricular, pre-auricular sinus, branchial cleft cyst, first branchial cleft

## Abstract

Two patients presented with fluctuant areas inferior to the pinna. The first required numerous procedures and investigations before a correct diagnosis was obtained. However, with awareness of this condition, the subsequent patient was quickly identified and managed appropriately. First branchial cleft abnormalities are uncommon, however, present with common symptoms. Their location and characteristics in paediatric patients is key to having it in the differential diagnosis. Consideration of this condition by ENT surgeons is key to prevent multiple invasive and futile operations in our paediatric cohort.

## Introduction

First branchial cleft abnormalities are rare and often misdiagnosed [1]. Patients commonly undergo multiple incision and drainage procedures prior to obtaining the correct diagnosis and thus the correct surgery [1]. With an average delay between first symptoms and successful treatment of three and a half years, more needs to be done to highlight the pathology to ENT surgeons [2].

Due to their congenital aetiology, they most commonly present in the paediatric population and can have variable locations but frequently occur in the retroauricular, parotid, submandibular or suprahyoid regions within an area described as Poncet’s triangle [2-4]. Poncet’s triangle has its apex at the external auditory canal (EAC) and base between chin and midpoint of hyoid bone with the two remaining sides joined from EAC to chin and from EAC to greater cornu of hyoid [2,4]. They most commonly affect females and are left-sided [5]. They can either be a cyst (no cutaneous connection), a sinus (one cutaneous connection), or a fistula (more than one cutaneous connection). Furthermore, they can present with otological symptoms such as otorrhoea with an intact tympanic membrane due to a fistula opening into the floor of the EAC [6,7]. First branchial cleft abnormalities are commonly misdiagnosed as a pre-auricular pit. However, these are distinct diagnoses which occur anterior to the tragus or helical root [7].

First branchial cleft abnormalities were classified by Work based on histology and embryology. Type one is ectodermal and is duplication of membranous auditory canal whereas type two is duplication abnormalities of membranous EAC and pinna and contains both ectoderm and mesoderm [6,8]. Other classification systems exist such as Arnot and Oslen, however, are less commonly used [6]. A recently proposed classification system based on MRI findings may be more appropriate for further studies as it may more accurately distinguish between patient groups [9]. Furthermore, although widely used, Work and Arnot classifications are not that useful clinically but are rather histological observations.

The article "First Branchial Cleft Anomalies: Awareness Is Key" was published in 2021. Journal: Cureus.

Diagnosis can be confirmed either by ultrasound or most commonly using MRI [6]. This allows the surgeon to plan appropriately and identify the risk of facial nerve damage due to the known variable relationship of the lesion to the facial nerve [6]. Complete excision is required to prevent recurrence and most excision is via a superficial parotidectomy approach [1-3,10].

## Case presentation

Case 1

A two-and-a-half-year-old girl was referred in to the ENT clinic with a tender fluctuant area involving the pre-auricular and inferior aspect of the pinna with mildly raised inflammatory markers (c-reactive protein: 45). The patient had no significant medical or prenatal related history. The patient was diagnosed with a peri-auricular abscess and underwent an incision and drainage of the lesion under general anaesthesia. Intraoperatively, the EAC and tympanic membrane were normal, however, a left-sided peri-auricular abscess was drained with pus sent to histology and microbiology for microscopy, culture and sensitivity, and to test for acid-fast Bacilli (AFB). The wound was washed out with 0.9% saline and betadine and a bismuth iodoform paraffin paste (BIPP) dressing applied. The patient was sent home to complete a seven-day course of oral antibiotics. The BIPP dressing was removed two days later and appeared to have healed well.

The patient was seen two weeks after the initial procedure. Full re-accumulation of the abscess had occurred. Previous histology showed inflammatory granulation tissue and no growth was seen on microbiology with AFB negative. The patient underwent a further incision and drainage under general anaesthesia. The wound was noted to be discharging from the previous scar and thus the wound was opened up with the granulation tissue debulked and sent for histology which again showed only inflammatory granulation tissue. Despite good early healing, the parents reported having to change the dressing daily owing to high wound output. The patient was unfortunately lost to follow up but represented eight months later and on this occasion, the lesion was solely inferior to the pinna and was noted to have a communication with the EAC with discharge noted with an intact tympanic membrane. The patient underwent a further incision and drainage, however, in postoperative follow-up, a possible diagnosis of a first branchial cleft abnormality was considered and a referral was made to a paediatric ENT specialist centre. The patient had an MRI which confirmed the diagnosis showing a left pre-auricular cystic swelling with a thick-walled and mildly enhancing tract extending to the floor of the lateral bony EAC suggestive of a first branchial cleft cyst (Figure 1). The patient underwent an excision of the fistula via a parotidectomy approach.

The article "First Branchial Cleft Anomalies: Awareness Is Key" was published in 2021. Journal: Cureus.

**Figure 1:** T2-weighted MRI showing thick-walled and mildly enhancing tract extending from lesion immediately anterior to the lobule of the pinna to the floor of the lateral bony external auditory meatus

Case 2

A two-year-old was referred to the paediatric team with a suspected infected insect bite approximately a month after case one. The lesion was left-sided and inferior to the pinna approximately over the angle of the mandible. The patient had a history of infantile eczema but no longer required treatment. Upon review, the lesion was not erythematous or painful and there were no active signs of infection. An outpatient ultrasound was organised to identify the cause. The scan showed a collection of debris subcutaneously adjacent to the left parotid (Figure 2A). It was felt that the appearances suggested an infected lymph node that initially started as an abscess but had then progressed into a collection of debris. On follow up in the paediatric clinic, the lesion had further increased in size, however, had otherwise not changed in character. Without spontaneous resolution, an otolaryngology consult was sought. On review, the tympanic membrane and EAC were clear, however, an indurated defect with discharge was seen in left Poncet’s triangle. A specific ultrasound request to look for evidence of a branchial cleft cyst was ordered which on this occasion found features consistent with a first branchial cleft cyst in the left upper neck posterolateral to the angle of the mandible and extending into the tail of the left parotid (Figure 2B). The patient was referred to a specialist centre for excision of the lesion.

**Figure 2:** A: Ultrasound of the left neck showing debris subcutaneously adjacent to left parotid. B: Ultrasound of the left neck showing lenticular shaped collection with a hypoechoic tract extending from the superficial lesion into the posterior aspect of tail of left parotid salivary gland

## Discussion

Both of these cases show the need for awareness and understanding of branchial cleft abnormalities. The initial patient presented with signs suggestive of an abscess, however, despite increasing evidence such as negative microbiological samples, high wound output, and lack of temperature or other signs of infection, diagnostic overshadowing occurred leading to repeated procedures that did not address the root cause of the patients’ symptoms.

The article "First Branchial Cleft Anomalies: Awareness Is Key" was published in 2021. Journal: Cureus.

The patient underwent four incision and drainage procedures prior to having the appropriate surgery. This is similar to previous case reports of these presentations [1]. They both presented with signs similar to those expected for a first branchial cleft cyst [6,7], however, with the second case, prompt diagnosis was made due to the clinician familiarity and awareness of the diagnosis.

Branchial cleft abnormalities are uncommon. However, they can present with symptoms familiar to many clinicians with the right experience [3]. First branchial cleft abnormalities should be considered with a patient presenting with either a cyst, sinus, or fistula in Poncet’s triangle or chronic/recurrent upper neck infections, especially if ipsilateral otological disease [2,4,7]. Patients can present with an infected first branchial cleft cyst causing an abscess, however, all suspected abscesses in this area should be thoroughly investigated. If a branchial cleft abnormality is present, surgery should be avoided if possible, as scarring from multiple procedures has been shown to increase the risk of facial nerve palsy during subsequent excision [7] and the rate of recurrence [10]. Sinuses and fistulas tend to be diagnosed earlier due to obvious skin openings and discharge and are more likely to become infected and thus present to healthcare services earlier [10]. Both these cases initially presented as cysts and thus likely contributed to the delay in diagnosis. Evidence of purulent discharge from the EAC upon pressure in the neck shows a connection between the lesion and the EAC and concurrent tympanoplasty or canalplasty could be considered to correct the defect in these lesions [7].

Clinicians need to ensure diagnostic breadth and awareness of confirmation bias in consultations with patients. This is especially important in the paediatric patient group where uncommon congenital lesions can present in a similar manner to more common diagnoses. MRI is still the gold standard diagnostic modality and is required for operative planning, however, CT scan can also be used to define the anatomy of the lesion in relation to surrounding structures preoperatively [3,10]. Infants commonly require sedation for CT or MRI, however, ultrasound is usually well tolerated [10]. A focused ultrasound, such as in the second case, is a useful tool in quickly identifying the diagnosis. Sonographic features of branchial cleft abnormalities can include lesions with a smooth outline and uniformly anechoic with posterior enhancement, however, their features have also been shown to be variable and therefore its value is inconsistent and can be operator dependent [10].

The article "First Branchial Cleft Anomalies: Awareness Is Key" was published in 2021. Journal: Cureus.

If feasible surgical excision should occur prior to infection of the lesion as this can distort surgical planes, and it makes successful excision more challenging [10]. Facial nerve monitoring should be used in all cases [1,3,7]. Standard parotidectomy incision and facial nerve dissection is required, however, dissection rarely extends further than 1-2 cm past the division of the facial nerve [1-3,10]. Recurrence rates are variable and dependent on number of preoperative procedures and infections, and the ability to fully excise the lesion, however, one report put it at 8% [10].

## Conclusions

The authors describe two cases of branchial cleft abnormalities. The patients had similar presentations, both consistent with the diagnosis, however, their patient journey was markedly different due to clinician awareness of the condition. MRI and ultrasound are both useful diagnostic aids. ENT clinicians should have a strong suspicion of branchial cleft abnormalities in any paediatric patient with a discharging lesion presenting in Poncet’s triangle.

## References

[1] Magdy EA, Ashram YA (2013). First branchial cleft anomalies: presentation, variability and safe surgical management. Eur Arch Otorhinolaryngol.

[2] Triglia JM, Nicollas R, Ducroz V, Koltai PJ, Garabedian EN (1998). First branchial cleft anomalies: a study of 39 cases and a review of the literature. Arch Otolaryngol Head Neck Surg.

[3] Goff CJ, Allred C, Glade RS (2012). Current management of congenital branchial cleft cysts, sinuses, and fistulae. Curr Opin Otolaryngol Head Neck Surg.

[4] Tham YS, Low WK (2005). First branchial cleft anomalies have relevance in otology and more. Ann Acad Med Singap.

[5] D’Souza AR, Uppal HS, De R, Zeitoun H (2002). Updating concepts of first branchial cleft defects: a literature review. Int J Pediatr Otorhinolaryngol.

[6] Kumar R, Sikka K, Sagar P, Kakkar A, Thakar A (2013). First branchial cleft anomalies: avoiding the misdiagnosis. Indian J Otolaryngol Head Neck Surg.

[7] Shinn JR, Purcell PL, Horn DL, Sie KC, Manning SC (2015). First branchial cleft anomalies: otologic manifestations and treatment outcomes. Otolaryngol Head Neck Surg.

[8] Work WP (1972). Newer concepts of first branchial cleft defects. Laryngoscope.

[9] Liu W, Chen M, Liu B, Zhang J, Ni X (2021). Clinical analysis of type II first branchial cleft anomalies in children. Laryngoscope.

[10] Schroeder JW Jr, Mohyuddin N, Maddalozzo J (2007). Branchial anomalies in the pediatric population. Otolaryngol Head Neck Surg.

